# Differences in the expression profiles of claudin proteins in human nasopharyngeal carcinoma compared with non-neoplastic mucosa

This article has been retracted.

**DOI:** 10.1186/s13000-018-0685-0

**Published:** 2018-02-05

**Authors:** Xiaowei Zhang, Haiming Wang, Qian Li, Yunpeng Liu, Peiqing Zhao, Tao Li

**Affiliations:** 1 Center for Translational Medicine; Department of Spinal Surgery, Central Hospital of Zibo, Affiliated with Shandong University, Gongqingtuan Road 54Hao, Zibo, Shandong Province China; 2 Department of General Surgery, People’s Hospital of Linzi District, Affiliated with Binzhou Medical College, Shandong Province, China; 3 Department of Spinal Surgery, Central Hospital of Zibo, Affiliated with Shandong University, Zibo, Shandong Province China; 4 Department of Thoracic Surgery, the First Hospital of Jilin University, Changchun, Jilin China

**Keywords:** Tight junction, Claudin-2, Claudin-5, Claudin-8, Claudin-9, Nasopharyngeal carcinoma

## Abstract

**Background:**

Several studies have suggested that claudin proteins, which are the main components of tight junction structures, are related to the regulation of cell polarity and cell differentiation.

**Method:**

To explore the expression profiles of the tight junction proteins claudin-2, − 5, − 8 and − 9 in nasopharyngeal carcinoma, IHC (immunohistochemical analysis), Western blot and real-time PCR were used to detect the expression profiles of these claudin proteins in nasopharyngeal carcinoma tissues and in non-neoplastic mucosal tissues.

**Results:**

According to our study, the expression levels of claudin-2 and claudin-5 were reduced, while the expression of claudin-8 was increased in nasopharyngeal carcinoma tissues in comparison with non-neoplastic mucosal tissues. Correlations between claudin-2 and -5 expression and metastatic progression in nasopharyngeal carcinoma patients were also found.

**Conclusion:**

In summary, our research reveals distinct expression profiles of claudin-2, − 5 and − 8 in non-neoplastic mucosal tissues and nasopharyngeal carcinoma tissues. In addition, the expression of these claudin proteins was highly correlated with metastatic progression and prognosis in patients with nasopharyngeal carcinoma and had predictive value for the metastasis and survival of nasopharyngeal carcinoma patients.

## Background

At present, studies have revealed that tight junctions (TJs), which are composed of a network of strands that encircle the cells, have crucial functions in the formation of epithelial cell sheets which overlap over the external and internal surfaces of organs [1]. Considering that the majority of cancers are derived from the epithelium [2], the cellular processes that mediate the acquisition of a tumorigenic phenotype of epithelial cells have become an important area of scientific research [3, 4]. Recently, the destruction of the structure of tight junctions (TJs) has become a well-accepted factor that endows transformed epithelial cells with metastatic capability [5]. Recent research has reported that TJs not only have a vital effect on cell polarity but that they also affect cell proliferation, metastasis and invasion. The destruction of the structure of TJs was revealed to lead to the disruption of epithelial cell cohesion and the promotion of epithelial cell invasiveness [5–7].

The claudin proteins, which are the primary molecules that participate in TJs, include 27 integral membrane proteins [8–10]. In most tissues, the combination of multiple claudin proteins leads to the formation of TJs through homotypic or heterotypic interactions, or through their interaction with other TJ proteins [11, 12]. Recently, it was suggested that the expression profiles of claudin proteins varied among different tissue types. Additionally, the claudin proteins were reported to interact with other tight junction proteins and to participate in cell signaling pathways through a PDZ domain in the C-terminus within the cytoplasm [8, 13–17],which suggested that the functions of claudin proteins may be highly tissue-specific and may depend on the active molecular pathway in epithelial cells abnormal expression of claudin proteins may have a particular role in cancer progression [18]. Thus, the objective of this study was to explore the expression profiles of claudins, which are tight junction molecules, in nasopharyngeal carcinoma and non-neoplastic mucosal tissues.

## Methods

### Patients

Sections were collected from 70 patients with nasopharyngeal carcinoma who were treated at the First Hospital of Jilin University between May 2004 and July 2010. The cases were selected based on the following criteria: pathologically confirmed diagnosis of nasopharyngeal carcinoma; no previous malignant disease or second primary tumor; and no history of radiotherapy and chemotherapy. All the nasopharyngeal carcinoma patients were graded and classified according to the International Union against Cancer (UICC) staging system. Histologically normal nasopharyngeal tissues were also obtained from patients with inflamed or enlarged tonsils that were found to be histologically non-neoplastic. The medical records of the patients were reviewed to determine the clinical and pathological characteristics.

### Immunohistochemistry

An immunohistochemical analysis was performed as previously described [19]. Sections were incubated with the rabbit anti-human claudin-2 antibody (ab53032), the rabbit anti-human claudin-5 antibody(ab15016), the rabbit anti-human claudin-8 antibody(ab183738), or the rabbit anti-human claudin-9 antibody (ab192398) diluted 1:450, 1:300, 1:350, and 1:400 at 4 °C overnight respectively. All these rabbit polyclonal antibodies were purchased from Abcam (Cambridge, MA, USA). Negative control sections were incubated with isotype antibodies.

### Western blotting

Western blotting was used to detect the expression of claudin proteins in the 12 human nasopharyngeal carcinoma tissues and non-neoplastic mucosae, which were randomly selected from the 70 samples of nasopharyngeal carcinoma tissues and homologous non-neoplastic mucosal tissues. Tissue lysates were prepared from each nasopharyngeal carcinoma tissues and non-neoplastic mucosae, and protein concentration was determined using BCA Protein Assay Kit (Pierce Chemical Co., Rockford, Illinois, USA). Twenty micrograms of total proteins were separated on 10% SDS-PAGE and then transferred onto nitrocellulose membrane. Western blot was performed as previously described [20]. Briefly, the membranes were probed overnight at 4 °C with the primary antibody (anti-claudin-2, 1:1000; anti-claudin-5, 1:1000; anti-claudin-8, 1:1000; anti-claudin-9, 1:1000; Abcam, San Francisco, CA, USA), and these claudin proteins were detected at about 22 kDa in the gel.

### Real-time PCR for the detection of claudin mRNA

RNA was isolated from frozen specimens using TRIzol reagent (Sangon, Shanghai, China) according to the manufacturer’s instructions. One microgram RNA was reverse-transcribed using M-MLV Kit (TAKARA, Shiga, Japan) and random 9-mer primers (TAKARA). Semiquantitative PCR were conducted using 50 ng of reverse-transcribed cDNA and 0.4 μM of each primer in a final reaction volume of 20 uL containing 1 × PCR master Mix (TAKARA). Typical real-time PCR reactions were performed as previously described [20]. The relative expression was based on the expression ratio of a target gene versus that of GAPDH. The primers used were as follows: claudin-2 forward primer (5′-CCAACCTCAGCCAGAGAGAGG-3′) and claudin-2 reverse primer (5′-TCCCCAAACCCACTAATCACA-3′); claudin-5 forward (5′-CCTTCATCGGCAACAGCATC-3′) and reverse (5′-CGTACACCTTGCACTGCATC-3′); claudin-8 forward (5′-GTCAGGTCTGTGTTCCATG-3′) and reverse (5′-TGACACCGC CAATGATGC-3′′); claudin-9 forward (5′-ATGGTAGCCACTTGCCTTC-3′) and reverse (5′-TTAGACATGGGCACTCTTGG-3′); and glyceraldehyde phosphate dehydrogenase (GAPDH) forward (5’-AACGTGTCAGTCGTGGACCTG-3′) and reverse (5’-AGTGGGTGTCGCTGTFGAAGT-3′).

### Criteria for the positive expression of claudin proteins in nasopharyngeal tissues

The staining and scoring of the claudin protein expression levels were classified semiquantitatively based on the total combined scores of the percentage of positively stained tumor cells together with the staining intensity [21]. A tumor was scored as ‘0’ if < 5% of tumor cells stained positive, ‘1’ if 5–30% of cells were positive, ‘2’ if 30–50% of cells were positive and ‘3’ if > 50% of cells were positively stained. The staining intensity was scored as ‘0’ if no cells were stained or if only weak staining was present, ‘1’ if moderate staining was present, and ‘2–3’ in cases of strong staining. The final score of the claudin protein expression was defined as ‘low claudin expression’ if the sum of the positivity score and the staining intensity score was 0–1, and ‘high claudin expression’ if the sum was 2–3. In each case, at least five different areas of the tumor were examined, and the mean of the results was used as the final expression score.

### Follow-up

Patients were followed-up to 59 months to evaluate metastasis and to determine survival. Survival time was calculated as the time from the beginning of diagnosis to the time of death or loss to follow-up. By the end of June 2015, the living status of all patients had been confirmed though either an outpatient basis or telephone interview.

### Statistical analysis

All data were presented as the mean ± SD. Origin 7.5 laboratory data analysis software (Origin Lab Corp, Northampton, MA, USA) and image processing software (Image-Pro Plus6.0) were utilized to quantify the data. The prognostic significance and value was explored by the Chi-square test/Chi-Square Goodness-of-Fit Test and a *t*-test was used to explore the significance of the differences between two groups. Survival was analyzed by the Kaplan-Meier method and compared by log-rank tests.

## Results

### The expression of claudin-2, − 5 and − 8 varied between nasopharyngeal carcinoma tissues and normal mucosae

The expression of claudin proteins was explored in the membranes of nasopharyngeal carcinoma tissues and non-neoplastic mucosal tissues. As shown in Table 1, a high expression of claudin-2 was seen in 24.3% (17/70) of nasopharyngeal carcinoma tissues and in 45.7% (32/70) of mucosal tissues (Fig. 1a, b). High claudin-5 expression was seen in 30.0% (21/70) of nasopharyngeal carcinoma tissues and in 60.0% (42/70) of mucosal tissues (Fig. 1c, d). Membranous expression of claudin-8 was seen in 52.8% (37/70) of nasopharyngeal carcinoma tissues and in 21.4% (15/70) of mucosal tissues (Fig. 1e, f). The expression of claudin-9 in the cell membrane was low in nasopharyngeal carcinoma tissues (20/70) and in mucosal tissues (22/70) (Fig. 1g, h). These data revealed that the expression of claudin-2 and claudin-5 was decreased, while that of claudin-8 was increased in nasopharyngeal carcinoma.

**Table 1:** Expression of claudin-2 and claudin-5 and the clinicopathological characteristics in nasopharyngeal carcinoma patients

Item	*n*	claudin-2 (high)	claudin-2 (low)	*P*	*n*	claudin-5 (high)	claudin-5 (low)	*P*
Nasopharyngeal carcinoma tissue	70	17	53	< 0.01	70	21	49	< 0.01
Mucosae	70	32	38		70	42	28	
Age (years)								
≤60	37	10	27	0.896*	37	9	28	0.364*
> 60	33	7	26		33	12	21	
Histological grade								
Well-differentiated	31	9	22	0.472*	31	10	21	1.000*
Moderately and poorly differentiated	39	8	31		39	11	28	
Lymph node metastasis								
–	21	6	15	0.792*	21	4	17	< 0.05
–	49	11	38		49	17	32	
Ki67								
+	22	5	17	1.000*	22	6	16	1.000*
–	48	12	36		48	15	33	
Clinical stage								
I~II	27	7	20	0.364*	27	5	22	< 0.01
III~IV	43	10	33		43	16	27	

^*^No statistical significance was found with the Chi-square test/Chi-Square Goodness-of-Fit Test

**Fig. 1:** Membrane expression of claudin proteins in human nasopharyngeal carcinoma and non-neoplastic mucosae. **a**, claudin-2 expression in tissues: non-neoplastic mucosal tissues (left) and in human nasopharyngeal carcinoma tissue (right) **(b)**. **c**, expression of claudin-5 was detected in non-neoplastic mucosal tissues (left) compared with human nasopharyngeal carcinoma tissues (right) **(d). e**, claudin-8 expression in non-neoplastic mucosal tissues a (left) compared with human nasopharyngeal carcinoma tissues (right) **(f). g**, claudin-9 expression was detected in non-neoplastic mucosal tissues (left) and in human nasopharyngeal carcinoma tissues (right) **(h)** (400×)

As it displayed in Table 1, the expression of claudin-2 was not associated with age (*P* = 0.896), the expression of Ki67 (*P* = 1.000), histological grade (*P* = 0.472), clinical staging (*P =* 0.364) or lymph node metastasis (*P* = 0.792). The expression of claudin-5 was not associated with age (*P* = 0.364), histological grade (*P =* 1.000), or expression of Ki67 (*P =* 1.000), whereas it was associated with lymph node metastasis (*P* < 0.05) and clinical staging (*P* < 0.01). As shown in Table 2, the expression of claudin-8 was not related to age (*P* = 0.846), Ki67 expression (*P* = 0.472), histological grade (*P* = 1.000) or clinical staging (*P* = 1.000), whereas it was positively related with lymph node metastasis (*P* < 0.01). Patients with metastases were more likely to be negative for claudin-2 and -5 and were more likely to be positive for claudin-8 expression than were patients with non-metastatic disease. The expression of claudin-9 in nasopharyngeal carcinoma tissues was not noticeably different from that in histologically normal non-neoplastic mucosal tissues (Fig. 1g, h) (*P* = 1.000). Moreover, the expression of claudin-9 was not related to age (*P* = 1.000), histological grade (*P* = 1.000), expression of Ki67 (*P* = 0.486), lymph node metastasis (*P* = 1.000) and clinical staging (*P* = 0.162) (Table 2), these data revealed that claudin-9 expression in nasopharyngeal carcinoma was not noticeably different from that in non-neoplastic mucosa.

**Table 2:** Expression of claudin −8 and claudin −9 and the clinicopathological characteristics in nasopharyngeal carcinoma patients

Item	*n*	claudin-8 (high)	claudin-8 (low)	*P*	*n*	claudin-9 (high)	claudin-9 (low)	*P*
Nasopharyngeal carcinoma tissue	70	37	53	< 0.01	70	20	50	1.000*
Mucosae	70	15	55		70	22	48	
Age (years)								
≤60	37	21	16	0.846*	37	11	26	1.000*
> 60	33	16	17		33	9	24	
Histological grade								
Well-differentiated	31	22	10	1.000*	31	9	22	0.736*
Moderately and poorly differentiated	39	45	23		39	11	28	
Lymph node metastasis								
–	21	16	5	< 0.01	21	8	13	1.000*
–	49	21	28		49	12	37	
Ki67								
+	22	9	13	0.472*	22	9	13	0.486*
–	48	28	20		48	11	37	
Clinical stage								
I~II	27	14	13	1.000*	27	6	21	0.162*
III~IV	43	23	20		43	14	29	

^*^No statistical significance was found with the Chi-square test/Chi-Square Goodness-of-Fit Test

### Expression of claudin proteins in **mucosal and nasopharyngeal carcinoma tissues**

Semiquantitative immunoblotting was used to compare and estimate the statistical differences in the expression of claudin proteins in mucosal and nasopharyngeal carcinoma tissues. According to the scanned image, the expression levels of claudin-2 and claudin-5 were significantly down-regulated in nasopharyngeal carcinoma tissues compared with non-neoplastic mucosal tissues (Fig. 2a, b). The expression of claudin-8 was up-regulated in nasopharyngeal carcinoma tissues compared with non-neoplastic mucosal tissues (Fig. 2c). The difference in claudin-9 expression was not statistically significant between nasopharyngeal carcinoma tissues and mucosal tissues (Fig. 2d). The statistical differences in the expression of the claudin proteins are shown in Fig. 2e.

**Fig. 2:** Expression of claudin proteins in human nasopharyngeal carcinoma and non-neoplastic mucosae. Semiquantitative immunoblotting was used to estimate statistical differences in the expression of claudin proteins in 12 human nasopharyngeal carcinoma tissues and non-neoplastic mucosae. The semiquantitative measurements are expressed as the mean standard deviation and as percent changes from an internal reference sample. **a**) claudin-2 expression; **b**) claudin-5 expression; **c**) claudin-8 expression; **d**) claudin-9 expression; **e**) Histograms. *P < 0.05 and **P < 0.01 compared with non-neoplastic mucosae

### Expression of claudin mRNA in **nasopharyngeal carcinoma and mucosae**

Real-time PCR was performed to determine the statistical differences in the mRNA expression of claudin proteins in mucosal and nasopharyngeal carcinoma tissues. As shown in Fig. 3, the expression levels of claudin-2 and claudin-5 were significantly down-regulated in nasopharyngeal carcinoma tissues compared with mucosal tissues. The expression of claudin-8 mRNA was up-regulated in nasopharyngeal carcinoma tissues compared with non-neoplastic mucosae. The difference in claudin-9 mRNA expression between nasopharyngeal carcinoma tissues and non-neoplastic mucosal tissues was not statistically significant. These results correspond to the results obtained by immunoblotting.

**Fig. 3:** mRNA expression levels of claudins in human nasopharyngeal carcinoma and non-neoplastic mucosae. Real-time PCR analysis of claudin expression in 12 human nasopharyngeal carcinoma tissues and non-neoplastic mucosae. *P < 0.05 and **P < 0.01 compared with non-neoplastic mucosae

### Claudin-2 and claudin-5 were concurrently expressed in nasopharyngeal carcinoma tissues and non-neoplastic mucosal tissues.

In addition, the relevance of claudin-2 and claudin-5 expression was also explored. As shown in Tables 3 and 4, the expressions of claudin-2 and claudin-5 were found to be relevant in nasopharyngeal carcinoma tissues and non-neoplastic mucosal tissues.

**Table 3:** Correlation between the expression of claudin-2 and claudin-5 in nasopharyngeal carcinoma tissues

Item	claudin-5 (high)	claudin-5 (low)	φ*	*P*
claudin-2 (high)	10	11	0.874	< 0.01
claudin-2 (low)	7	42

**Table 4:** Correlation between the expression of claudin-2 and claudin-5 in non-neoplastic mucosae

Item	claudin-5 (high)	claudin-5 (low)	φ*	*P*
claudin-2 (high)	26	6	0.742	< 0.01
claudin-2 (low)	16	22		

### Clinical correlations and survival

Patients with claudin-2-positive primary tumors had a significantly longer survival (median 49.23 ± 2.67 months) than those with claudin-2-negative tumors (median 36. 31 ± 5.43 months) (*P* = 0.016; Fig. 4a). Similarly, patients with claudin-5-positive primary tumors had a significantly longer survival (median 48.61 ± 4.02 months) than those with claudin-5-negative tumors (median 37.12 ± 3.14 months; *P* = 0.012; Fig. 4b). Patients with claudin-8-positive primary tumors had a significantly shorter survival (median 36.97 ± 2.72 months) than patients with claudin-8-negative tumors (median 48. 93 ± 3.72 months) (*P* = 0.002; Fig. 4c). Patients with claudin-9-positive primary tumors had a significantly shorter survival (median 42.21 ± 3.12 months) than those with claudin-9-negative tumors (median 42. 68 ± 2.34 months) (*P* = 0.549; Fig. 4d). Patients with tumors that were positive for claudin-2 and claudin-5 proteins had a significantly longer survival than those whose tumors were negative for these two proteins, while patients with tumors that were positive for claudin-8 protein expression had a significantly shorter survival than those whose tumors were negative for this protein.

**Fig. 4:** The correlation between the expression of claudins and survival. Kaplan-Meier analysis were used for survival analysis in nasopharyngeal carcinoma patients A: Claudin-2 Curve; B: Claudin-5 Curve; C: Claudin-8 Curve; D: Claudin-9 Curve

## Discussion

The determination of the molecular mechanisms for TJ-based regulation of the microenvironment of epithelial cells is of great value to cancer research [5, 22]. Increasing evidence has verified that the loss of the structure of TJs in tumor progression is a mechanism in the process of cancer metastasis [23, 24]. The loss of tight junction structure caused by aberrant expression of claudin proteins has been suggested to be of extreme importance in the promotion of the diffusion of nutrients and other factors that are necessary for the survival and proliferation of cancer cells [25, 26]. Recent research has revealed that the expression of claudin proteins is frequently altered in various cancers. The abnormal expression profile of claudin proteins in tumor cells is coupled with the loss of cell polarity [27]. This was demonstrated in a recent study, which suggested that the expression of claudin-1 was down-regulated in pancreatic cancer cells and that re-expression of claudin-1 reduced the invasive ability of these cells [27, 28]. Similarly, it was revealed that the expression of claudin-8 was down-regulated in head and neck cancer and invasive breast cancer [29].

The differential regulation of claudin proteins in various cancer types represents an opportunity to determine the mechanism of different therapeutic responses [25, 30–32]. Hsueh C have reported the expression of claudin- 1, − 4 and − 7 in nasopharyngeal carcinoma patients, and revealed that claudin-4 and claudin-7 may be a novel biomarker for the prediction of distant metastasis and unfavorable prognosis in nasopharyngeal carcinoma [33]. Meanwhile, Lee JW has also reported that the upregulated claudin-1 expression confers resistance to cell death of nasopharyngeal carcinoma cells [34]. These result suggested that the expression profiles of claudin proteins varied in nasopharyngeal carcinoma. In the present study, IHC, semiquantitative immunoblotting and real-time PCR were used to compare and estimate statistical differences in the expression of claudin proteins in mucosal and in nasopharyngeal carcinoma tissues. Our data revealed that, compared with non-neoplastic mucosa, the expression levels of claudin-2, and claudin-5 were down-regulated, while the expression level of claudin-8 was up-regulated in nasopharyngeal carcinoma. In view of the specificity of claudin expression profiles in human cancer, it has been revealed that claudin proteins may serve as useful molecular markers for cancer diagnostics and the expression of claudin proteins can be used as a prognostic indicator, as the loss of claudin-1 has been suggested to be correlated with a poor prognosis in patients with stage II colon cancer [35]. Moreover, it was also reported that the expression of claudin-8 was an independent prognostic factor for the recurrence of hepatocellular carcinoma after curative hepatectomy [36]. In our study, correlations between the expression of claudin-5 and claudin-8 and lymph node metastasis were also observed, which revealed that the expression levels of claudin-5 and claudin-8 also have the potential to be established as prognostic indicators in patients with nasopharyngeal carcinoma. In addition, claudin-2 and claudin-5 were concurrently expressed in the mucosae and in nasopharyngeal carcinoma tissues, which revealed that claudin-2 and claudin-5 may jointly participate in the composition of tight junction structure in nasopharyngeal tissues. Moreover, patients with tumors that were positive for claudin-2 and claudin-5 protein expression had a significantly longer survival than those with negative tumors, while those with tumors that were positive for claudin-8 protein expression had a significantly shorter survival than those with negative tumors. This suggested that the expression of claudin-2, − 5 and − 7 might be a predictor of the development of metastases as well as a useful prognostic factor in nasopharyngeal carcinoma. In view of these observations in our study, we propose that patients should be screened after surgery for the expression of these claudin proteins. Given the correlation of the expression of these claudin proteins and survival, these proteins may represent novel tumor markers and therapeutic targets.

Given that the changes in claudin expression can be diverse and tissue-specific, numerous studies have investigated the functional correlation between these alterations in the expression of specific claudin proteins and tumorigenic growth and progression [19, 23, 37]. These studies have revealed that alterations in the expression of claudin proteins have crucial effects on the malignant phenotype of tumor cells [25, 38, 39]. For instance, in one study, claudin-1 remarkably inhibited the invasive and metastatic ability of breast cancer cells [40–42]. Conversely, the up-regulation of claudin-1 has been suggested to promote the invasive ability of colon cancer cells [43]. It was also shown that the positive feedback regulation between claudin-1 and the Wnt-signaling pathway plays a vital role in colon tumorigenesis. Moreover, the up-regulation of claudin-1 has also been reported to contribute to EMT through the c-Abl/Raf/Ras/ERK signaling pathway in hepatocellular carcinoma cells [43, 44]. In conclusion, these studies revealed that alterations in the expression of claudin proteins are associated with tumorigenic growth and progression [45, 46]. However, at present, few studies have examined the functional association between nasopharyngeal carcinogenesis and alterations in claudin protein expression [47–50]. In the future, we will address the specific mechanism that is responsible for our observations on how alterations in claudin protein expression affect the malignant and oncogenic phenotype of nasopharyngeal carcinoma.

## Conclusion

In summary, our present data inferred that the expression of claudin-2, − 5 and − 8 was altered between human non-neoplastic mucosa and nasopharyngeal carcinoma tissue and that their expression was correlated with lymph node metastasis.

## Abbreviation

CLDNs: claudins
IHC: **I**mmunohistochemical analysis
TJ: **T**ight junction
